The article "Adseverin knockdown inhibits osteoclastogenesis in RAW264.7 cells" was retracted in 2014. Reason: plagiarized text.

# Adseverin knockdown inhibits osteoclastogenesis in RAW264.7 cells

**DOI:** 10.3892/ijmm.2014.1941

**Published:** 2014-09-22

**Authors:** WENTING QI, YAN GAO, JUN TIAN, HONGWEI JIANG

**Affiliations:** Department of Operative Dentistry and Endodontics, Guanghua School and Hospital of Stomatology, Guangdong Provincial Key Laboratory of Stomatology, Sun Yat-sen University, Guangzhou, Guangdong 510055, P.R. China

**Keywords:** adseverin, RAW264.7, osteoclastogenesis, receptor activator of nuclear factor-κB ligand, actin filament

## Abstract

Osteoclastogenesis is a complex process that is highly dependent on the dynamic regulation of the actin cytoskeleton. Adseverin (Ads), a member of the gelsolin superfamily of actin-binding proteins, regulates actin remodeling by severing and capping actin filaments. The objective of the present study was to characterize the role of Ads during osteoclastogenesis by assessing Ads expression and using a knockdown strategy. Immunoblot analyses were used to examine Ads expression during osteoclastogenesis. A stable *Ads* knockdown macrophage cell line was generated using a retroviral shRNA construct. Osteoclast differentiation was morphologically examined via cell staining with osteoclast specific markers and light microscopy. The results showed that Ads expression was significantly increased in response to receptor activator of nuclear factor-κB ligand during osteoclastogenesis, and Ads was highly expressed in mature osteoclasts. Ads-knockdown macrophages showed major osteoclastogenesis defects, most likely caused by a pre-osteoclast fusion defect. These results indicate that Ads deficiency in monocytes inhibits osteoclastogenesis. Thus, in future studies it could be noteworthy to investigate the function of Ads in bone marrow monocytes during osteoclastogenesis.

## Introduction

Bone resorption is a pathological process associated with chronic periradicular periodontitis. Osteoclasts are the main cell type responsible for carrying out bone resorption. They are large, multinucleated cells that originate from the fusion of monocyte/macrophage lineage osteoclast precursors (1–3). Receptor activator of nuclear factor-κB ligand (RANKL) and macrophage colony stimulating factor (M-CSF) are significant factors for the fusion and differentiation of these precursors into mature osteoclasts. RANKL binds to its receptor, RANK, and induces osteoclast differentiation and activation via intracellular nuclear factor-κB (NF-κB) signaling. M-CSF plays a role in osteoclast precursor survival and proliferation. RANKL-induced osteoclast formation can be inhibited by osteoprotegerin (OPG), which acts as a decoy receptor for RANKL (4,5).

The actin cytoskeleton is responsible for a number of the structural and functional properties of osteoclasts. Dynamic changes in actin filament architecture are critical for pre-osteoclast motility, adhesion (6) and vesicle trafficking during cell fusion and osteoclast formation processes (7). Actin remodeling is involved in these physiologically significant processes, which is determined or regulated by a large number of actin-binding proteins, as well as by small Ras superfamily GTPases and actin-related proteins (8–11). *In vitro* studies revealed that gelsolin is one of the proteins regulating actin filament assembly dynamics. Gelsolin regulation of actin dynamics is calcium-dependent and occurs by severing preexisting filaments, capping the (+)-end of the newly generated filament following severing and nucleating actin filament assembly from monomers (12–15). These functional activities are frequent features among a family of proteins, including villin, adseverin, flightless and other gelsolin-like proteins, which have structural and functional homology to gelsolin (16–21).

Adseverin (Ads), also termed scinderin, is a member of the gelsolin family (22) and has been identified in several bovine tissues with secretory activity (23–25). Ads has also been noted in certain neuroendocrine and brain tissues, where it is expressed at low levels. Ads predominantly colocalizes with F-actin in bovine adrenal medulla chromaffin cells, whereas gelsolin is diffusely localized in these cells (26). Although gelsolin plays a key role in osteoclast function and motility (27–29), there are limited published studies regarding Ads expression in the monocyte/macrophage lineage or active osteoclasts. Additionally, its role in osteoclast formation and/or function has not been identified. Microarray analyses (30) have shown that the *Ads* gene is upregulated during osteoclastogenesis (OCG) and is highly expressed in mature osteoclasts. In the present study, *Ads*-knockdown was reported to inhibits OCG in RAW264.7 *in vitro*.

## Materials and methods

### Cell culture and in vitro OCG

OCG in RAW264.7 cells (passages 5–15; American Type Culture Collection, Manassas, VA, USA) was initiated by plating 5×10^4^ cells into each well of an 8-chamber BD Falcon glass culture slide (BD Biosciences Discovery Labware, Bedford, MA, USA). The cells were incubated in 0.7 ml Dulbecco’s modified Eagle’s medium (DMEM; Life Technologies, Grand Island, NY, USA) supplemented with 10% fetal bovine serum (FBS) and 10% antibiotic/antimycotic solution (164 IU/ml penicillin G, 50 μg/ml gentamicin, and 0.25 μg/ml fungizone; Sigma-Aldrich, Oakville, ON, Canada). Once cells were plated in the dishes, sRANKL was added at a final concentration of 60 ng/ml. sRANKL was purified from *E. coli* BL21(DE3) competent cells (Agilent Technologies, La Jolla, CA, USA) transformed with pGEX-4T-1-sRANKL (kindly provided by Dr M.F. Manolson) using glutathione sepharose 4B resin (GE Healthcare, Piscataway, NJ, USA). All the incubations were performed at 37°C in 5% CO_2_ humidified air for 4 days. Culture media was changed and sRANKL was supplemented on the second day in culture.

### Transfection and time-lapse confocal microscopy

In order to visualize sub-cellular localization of Ads and F-actin as they assemble and disassemble, as well as podosome dynamics in living osteoclasts, RAW264.7 cells were seeded into 6-well plates with 25-mm coverslips (VWR International, Radnor, PA, USA) in each well. The cells were transiently cotransfected with pEGFP-Ads and pRFP-Lifeact using the FuGENE HD Transfection reagent according to the manufacturer’s instructions (version 11.0; Roche Applied Science, Madison, WI, USA). The transfected cells were incubated with sRANKL for 4 days. Time-lapse video and images were obtained using Leica confocal fluorescence microscopy (magnification, ×40; Leica Microsystems, Buffalo Grove, IL, USA).

### RNAi

The pSIREN-RetroQ-DsRed-Express vector (Clontech Laboratories, Inc., Mountain View, CA, USA) was used to knockdown *Ads* in RAW264.7 cells. Oligonucleotides (top, 5′-gatccAACAAATATGAGCGTCTGATTCAAGAGATCAGACGCTCATATTTGTTTTTTTTACGCGTg-3′; and bottom strand, 5′-aattcACGCGTAAAAAAAACAAATATGAGCGTCTGATCTCTTGAATCAGACGCTCATATTTGTTg-3′) targeting *Ads*, 5′-AACAAATATGAGCGTCTGA-3′ (ACGT Corp., Toronto, ON, Canada), were annealed and inserted into the vector. Non-silencing control luciferase shRNA (top, 5′-GATCCGTGCGTTGCTAGTACCAACTTCAAGAGATTTTTTACGCGTG-3′; and bottom strand, 5′-AATTCACGCGTAAAAAATCTCTTGAAGTTGGTACTAGCAACGCACG-3′) was used to generate a scrambled control RNAi vector. GP-293 pantrophic packaging cells were co-transfected with RNAi vectors and the pVSV-G envelope protein-packaging vector using the FuGENE HD transfection reagent according to the manufacturer’s instructions (Roche Applied Science). Transfected GP-293 cells were incubated at 37°C for three days, and the virus-containing supernatant was harvested and centrifuged to remove cells. Viral supernatants were treated for 30 min at room temperature with 65 U/ml benzonase to degrade residual cellular DNA. Viral supernatant was passed through a Millex-HA 0.45-μm syringe-driven filter unit and used to infect RAW264.7 macrophages. Infected RAW264.7 macrophages were incubated for three days at 37°C and sorted based on the dsRed signal during fluorescence-activated cell sorting (FACS). Sorted cells were subjected to limiting dilutions to obtain final dsRed-positive colonies. *Ads* expression was examined at the mRNA and protein levels. The *Ads*-knockdown clone with the lowest Ads protein expression was used in subsequent experiments (*Ads*-KD). Luciferase knockdown (*Luc*-KD) and uninfected RAW264.7 cells were used as controls.

### Tartrate-resistant acid phosphatase (TRAcP) staining

On day 4 in culture, the cells were washed gently twice with pre-warmed phosphate-buffered saline (PBS), fixed in 4% paraformaldehyde (PFA), and stained for TRAcP, a chemical osteoclast marker. Briefly, fixed cells were incubated for 30 min at 37°C in a solution of naphthol AS-BI phosphate and fast-red TR salt (Sigma-Aldrich, St. Louis, MO, USA) in 0.2 M acetate buffer (pH 5.2) containing 100 mM sodium tartrate (Sigma-Aldrich). TRAcP-stained cells were washed three times with PBS, counterstained for 10 min with 4′,6-diamidino-2-phenylindole (DAPI; Sigma-Aldrich; 0.165 μM in PBS containing 0.1% Triton^®^ X-100), and viewed using a Nikon Ellipse E1000 microscope (Nikon, Tokyo, Japan). TRAcP^+^-multinucleated cells containing ≥3 nuclei were categorized as osteoclasts. The number of TRAcP^+^ osteoclasts and nuclei within these osteoclasts were counted in 10 random fields of view. The fusion index [FI = (number of nuclei of total osteoclasts/nuclei of total cells) ×100%] was calculated for these cell lines.

### Migration versus fusion assays

To evaluate the effect of the initial cell seeding density on OCG, WT and knockdown cell lines were seeded at three initial seeding densities: 1×10^4^, 5×10^4^ and 1.0×10^5^ cells/well, for low, normal and high density, respectively. Day 4 cultures were fixed and stained with TRAcP as described. The degree of osteoclast formation was determined by viewing stained cells at magnification, ×200. Representative images were obtained using a PixeLINK camera (PixeLINK, Ottawa, ON, Canada).

### Fluorescent staining and quantification of actin ring structure

The cells were seeded on coverslips as described. On day 4, the cells were fixed with 4% PFA for 20 min, permeabilized with 0.1% Triton X-100 in PBS for 5 min, and saturated in 1% bovine serum albumin in PBS. Alexa 488-conjugated phalloidin was added for 30 min to stain F-actin. DNA was stained using DAPI. The cells were mounted using Fluoromount (Sigma-Aldrich). Osteoclast actin rings were visualized using a Leica confocal microscope and the total number of rings/slide was counted.

### Assessment of bone resorption in vitro

Monocytes were plated onto dentine discs (Osteosite Dentine Discs; Immunodiagnostic Systems Inc., Fountain Hills, AR, USA) in 96-well plates as previously described (31). On day 4, the cells were removed using 6% sodium hypochlorite (10 min incubation) and cotton swabs. Discs were rinsed with water and stained with 1% (w/v) toluidine blue in 0.5% sodium borate for 5 min, followed by washes in water. The number and area of resorption pits were measured using ImageJ software (National Institutes of Health, Bethesda, MD, USA). Results are expressed as the total area resorbed/dentine disc, the number of resorption pits, and the average resorption area/pit.

### NF-κB and c-jun activation assays

To evaluate whether the RANKL-RANK signaling axis is intact in *Ads*-knockdown cells, activation of the transcription factors, NF-κB and c-jun, was measured. Activation was defined by their translocation into the nucleus. Osteoclasts were cultured as described for 4 days in 8-well chamber slides, and NF-κB and c-jun localization was visualized by immunostaining using NF-κB and c-jun activation kits (Thermo Fisher Scientific, Inc., West Palm Beach, FL, USA) and fluorescence microscopy (magnification, ×20; Nikon Eclipse E1000).

### Western blot analyses

The cells were rinsed with cold PBS and lysed in RIPA buffer (Sigma-Aldrich) supplemented with 1X protease inhibitor cocktail (BD Pharmingen, San Diego, CA, USA) and 1 mM phenylmethylsufonylfluoride (PMSF). The lysates were cleared with 5 min centrifugation at 13,000 rpm at 4°C. Total protein concentrations were measured using the bicinchoninic acid protein assay kit (Pierce, Rockford, IL, USA). Heat-denatured protein samples (20 μg) were electrophoresed in 10% polyacrylamide gels. Following electrophoresis, gels were transferred to nitrocellulose filters (Amersham Pharmacia Biotech, Piscataway, NJ, USA). Filters were maintained overnight in the primary antibody in 5% skimmed milk powder/Tris-buffered saline/Tween-20 (TBST), washed three times with TBST, and incubated for 60 min at room temperature in horseradish peroxidase (HRP)-conjugated secondary antibodies/5% skimmed milk powder in TBST. Following three TBST washes, membranes were incubated with Western Lightning solution (Perkin-Elmer, Waltham, MA, USA), and the resulting chemiluminescence was exposed to film (Kodak, Rochester, NY, USA). The following primary antibodies were used: Rabbit anti-mouse Ads (a gift from Dr C. Svensson; 1:2,000), rabbit polyclonal anti-murine-gelsolin antibody (a gift from Dr C. McCulloch; 1:2,000 dilution), and monoclonal anti-actin (cloneAC-74, 1:8,000 dilution; Sigma-Aldrich). The secondary antibodies used were HRP-linked goat anti-rabbit immunoglobulin G (IgG) (1:4,000 dilution; Amersham Pharmacia Biotech) and sheep anti-mouse IgG-HRP (1:8,000 dilution; Amersham Pharmacia Biotech).

### Statistical analyses

Results are expressed as the mean ± standard deviation. Each experiment was performed in triplicate unless otherwise stated. Statistical analyses were performed using Student’s t-tests or multiple t-tests. P<0.05 was considered to indicate a statistically significant difference. All the statistical analyses were performed using the SPSS 12.0 statistical package (SPSS, Inc., Chicago, IL, USA).

## Results

### Ads protein is upregulated during OCG

Ads protein expression in RAW264.7 cells (Fig. 1) was measured using western blot analyses. Increased Ads protein expression was observed in RAW264.7 cells, along with cell differentiation in the late stage of OCG. Gelsolin protein expression was also examined. However, gelsolin protein expression remained constant during OCG.

### Ads plays a role in actin assembly and cytoskeleton regulation in sRANKL-stimulated RAW264.7 cells

Ads is a Ca^2+^-dependent filamentous actin severing and capping protein. Therefore, its expression may produce changes in F-actin content and distribution. In order to visualize the sub-cellular localization of Ads in pre-osteoclasts and mature osteoclasts, RAW264.7 macrophages were transiently cotransfected with pEGFP-*Ads* and pRFP-Lifeact. The *Ads* construct allowed visualization of the localization of exogenous *Ads* tagged at its C-terminus with GFP. Similarly, RFP-tagged lifeact, a 17 amino acid peptide that binds specifically to F-actin without interfering with actin dynamics (32), allowed visualization of the actin structures in osteoclast progenitors and mature osteoclasts. Under resting conditions, subplasmalemmal Ads appears as a continuous fluorescent ring. In unstimulated cells, F-actin and Ads colocalized at the subplasmalemmal region in continuous and intense rings of fluorescence. Upon sRANKL stimulation for 3 days, cortical F-actin and Ads fluorescent rings were disrupted at the periphery with dot-like podosome structures, indicating redistribution of Ads and F-actin disassembly (Fig. 2A). Scatterplots showed that the Ads and F-actin overlap coefficient decreased from 0.94 (without sRANKL) to 0.91 (with sRANKL) (n=5) (Fig. 2B). The time-lapse video showed Ads and F-actin colocalized in actin rings and appeared to have a role in actin ring assembly and cytoskeleton regulation in mature OCs (Fig. 2C).

### Ads is required for RANK-mediated osteoclast formation

In order to confirm the role of Ads in OCG, OCG from *Ads*-knockdown and *Luc*-knockdown cells was confirmed. OCG was almost completely blocked in *Ads*-knockdown cells (Fig. 3A). *Ads*-null osteoclast-like cells that formed were aberrant, stunted and stained weakly for TRAcP. These cells also had only one or two nuclei (Fig. 3C). There was a significant decrease in fusion efficiency in *Ads*-knockdown cells (FI =0) compared to control *Luc*-knockdown cells containing scrambled shRNA (FI =41.40%) and untransfected control RAW264.7 cells (FI =26.11%) (Fig. 3B).

### Defective fusion of Ads-knockdown cells is not rescued by increased cell seeding density

At low, normal and high densities, no osteoclasts were formed from *Ads*-knockdown cells (Fig. 4). As density increased, the control cells formed larger osteoclasts, whereas *Ads*-knockdown macrophages never formed osteoclasts with >3 nuclei. The results of cell seeding density rescue assays indicate a fusion defect in *Ads*-knockdown cells.

### Ads knockdown impaired RANKL-induced actin ring formation and bone resorption

Mature OCs possess a sealing zone that consists of a filamentous actin ring that is required for bone resorption, and these cells have clear margins (33). Therefore, the effect of *Ads* knockdown on actin ring formation and bone resorption was subsequently evaluated. *Luc*-knockdown cells formed ~50 actin rings/field with clear and dense margins (Fig. 5A), whereas *Ads*-knockdown cells never formed actin rings (Fig. 5C). *Luc*-knockdown cells were capable of resorbing the dentin disc substrate at significantly higher rates than *Ads*-knockdown cells (Fig. 5D and E). *Ads*-knockdown osteoclastic cultures had almost no multinucleated osteoclasts on the dentin disks, as well as extremely small and barely detectable resorption pits (Fig. 5B).

### Ads ablation is associated with impaired RANK signaling

RANK downstream signaling was evaluated using NF-κB immunostaining on day 4 in *Ads*-knockdown and *Luc*-knockdown cells. NF-κB was activated in *Luc*-knockdown osteoclasts only, as shown by its exclusive nuclear distribution (arrows). *Ads*-knockdown monocytes did not exhibit active NF-κB as shown by its cytoplasmic distribution. However, monocytes and osteoclasts in the two groups demonstrated activated nuclear c-jun, a transcription factor involved in RANK signaling associated with apoptosis (Fig. 6).

## Discussion

Ads is associated with the regulation of chondrocyte differentiation (34). Notably, 2,3,7,8-tetrachlorodibenzo-dioxin (TCDD) upregulated Ads gene and protein expression (35), which was dependent on the aryl hydrocarbon receptor (AhR) (36). Furthermore, low concentrations of TCDD and other AhR agonists stimulate OCG and bone resorption (37). Osteoclast differentiation is a two-step process: The osteoclastic commitment stage and cell-cell fusion stage. Pre-osteoclasts must migrate toward each other in a chemotactic manner. The close proximity of cells, along with RANKL-mediated activation of the RANK receptor, is believed to induce fusion competency via transcription and surface expression of fusion receptors. Subsequently, fusion-competent cells recognize and adhere to one another, which is followed by membrane attachment and fusion. By seeding *Ads*-knockdown and control cells at low, normal and high densities, it was observed that regardless of seeding density, *Ads*-knockdown macrophages did not form TRAcP-positive multinucleated osteoclasts compared to the control cells. Further evidence against the involvement of *Ads* during pre-osteoclast migration is the observation of pronounced cellular clumps or colonies in *Ads*-knockdown cultures seeded at low and normal densities (data not shown). Notably, in the present experiments, *Ads*-knockdown cells were inclined to detach from the flask. Additionally, jet wash assays confirmed this observation (data not shown), implying that impaired adhesive ability may contribute to *Ads*-knockdown migration and aggregation. Therefore, a fusion defect is the most likely cause of defective OCG in *Ads*-knockdown cells.

Osteoclastic cell-cell fusion is highly dependent on actin assembly, which is required for cell shape alterations and actin-regulated plasma membrane reorganization. The actin-binding protein, Ads, increases chromaffin cell actin filament depolarization and regulates the stability of the cortical actin cytoskeleton in a calcium-dependent manner (38,39). In airway goblet cells, Ads rearranges the apical actin caps that act as a physical barrier to secretion (40). These results strongly indicate that Ads is involved in the control of cortical actin networks. Thus, Ads may influence OCG by regulating cortical actin assembly during cell fusion.

The actin cytoskeleton provides an active driving force for cell-cell fusion by generating membrane protrusions that are necessary and sufficient to promote fusion mediated by fusogenic proteins (41). Extensive cytoskeletal reorganization occurs prior and subsequent to fusion in cultured pre-osteoclasts. Video visualization of the actin cytoskeleton in our experiments revealed dynamic changes in *in vitro* mouse osteoclast fusion.

In order to visualize the sub-cellular localization of Ads in live pre-osteoclasts and mature osteoclasts, RAW264.7 macrophages were transiently cotransfected with pGFP-*Ads* and pRFP-Lifeact. The data showed that treating these cells with sRANKL disrupted the cortical F-actin network and redistributed Ads. Osteoclasts are uniquely motile as they continue to resorb bone beneath one area of the cell undersurface, whereas another area simultaneously reorganizes and moves, dependent on the actin rings (42). As the present video data show, Ads strongly colocalized with F-actin in actin rings. Despite OCG, it appeared that Ads also plays an important role in active osteoclast motility and resorption.

OCG requires the differentiation cytokine RANKL to bind to its receptor RANK, resulting in the intracellular RANK-TRAF6 interaction and subsequent activation of the transcription factors, NF-κB and activator protein 1 (AP-1) (consisting of c-fos and c-jun). The results showed that *Ads* knockdown is associated with impaired RANK signaling. Signaling downstream of RANK was evaluated by NF-κB immunostaining on day 4 of OCG. Based on its exclusively nuclear distribution, NF-κB was activated only in *Luc*-knockdown control osteoclasts. The majority of sRANKL stimulated *Ads*-knockdown cells did not exhibit activated NF-κB, as shown by its cytoplasmic distribution. RANKL is a required differentiation factor in OCG and has a secondary role as an antiapoptotic factor whose action is mediated by the c-Jun N-terminal kinases/c-jun pathway (43). In addition, c-jun complements AP-1 activation upstream of nuclear factor of activated T-cells, cytoplasmic 1 (NFATc-1) (3). *Ads*-knockdown cells express active, nuclear localized c-jun. Thus, the present data indicate that *Ads* does not mediate survival signaling downstream of RANK, but is required in early stages where dynamic actin remodeling is crucial for preosteoclast fusion.

In conclusion, the present study demonstrates that Ads is expressed in monocytes undergoing RANKL-induced OCG *in vitro*. Additionally, when Ads expression is suppressed, osteoclast formation and resorption function in RAW264.7 cells decreased. These results indicate that Ads is an important regulator of OCG. In addition, it appears that Ads affects the cell fusion process by inhibiting NF-κB activation. Further studies using the *Ads*-knockout mouse model are required to characterize Ads function and its role in the bone marrow monocyte/macrophage lineage, as well as to determine how Ads expression affects bone metabolism.

## Figures and Tables

**Figure 1:** Expression of adseverin (Ads) and gelsolin in *Ads*-knockdown RAW264.7 cells and RAW264.7 cells stimulated with sRANKL for 4 days. (A) Expression of Ads, gelsolin, and β-actin in RAW264.7 cells on days 0, 1, 2, 3 and 4 after RANKL stimulation using western blot analyses. (B) Protein expression levels of Ads and gelsolin were analyzed by western blotting. β-actin was used as a loading control. Band values were quantified by densitometric analyses. Gelsolin was expressed at similar levels on days 0, 1, 2, 3 and 4. However, Ads expression increased after day 3. RANKL, receptor activator of nuclear factor-κB ligand.

**Figure 2:** Immunofluorescence images of adseverin (Ads) (green) and F-actin (red) proteins in RAW264.7 cells following sRANKL administration. (A) Ads and F-actin colocalization is shown by the overlap of signals, resulting in yellow staining. In unstimulated RAW264.7 cells, F-actin and Ads colocalized in continuous and intense rings of fluorescence at the subplasmalemmal region. Upon sRANKL stimulation for 3 days, cortical F-actin and Ads rings are disrupted at the periphery with dot-like podosome structures, suggesting redistribution of Ads and F-actin disassembly during osteoclastogenesis. (B) Colocalized pixels of yellow color are located along the diagonal of the scattergram. Scatterplots showed that the Ads and F-actin overlap coefficient decreased from 0.94 (without sRANKL) to 0.91 (with sRANKL) (n=5). (C) Time-lapse confocal microscopy video frame shows Ads and F-actin colocalized in actin rings, actin ring assembly and disassembly during filming in mature OCs, indicating that Ads plays a role in actin assembly and cytoskeleton regulation. RANKL, receptor activator of nuclear factor-κB ligand.

**Figure 3:** Adseverin (*Ads*)-knockdown RAW264.7 macrophages exhibit profound defects in osteoclastogenesis. Wild-type, luciferase and *Ads*-knockdown RAW264.7 macrophages (5×10^4^ cells) were seeded into 8-well chamber slides and stimulated for 4 days with 60 ng/ml sRANKL to induce osteoclastogenesis. Images of TRAcP-stained osteoclasts were obtained (magnification, ×200). To visualize the nuclei, the cells were stained with 4′,6-diamidino-2-phenylindole (DAPI). (A) In order to confirm the role of Ads in osteoclastogenesis (OCG), OCG from *Ads*-knockdown and *Luc*-knockdown cells was compared. OCG was almost completely blocked in *Ads*-knockdown cells. (C) Osteoclasts were defined as TRAcP^+^ multinucleated cells containing ≥3 nuclei. TRAcP^+^ osteoclasts were classified based on the number of nuclei (≥3, ≥5 or ≥10 nuclei) within these osteoclasts and counted in 10 random fields of view (FOVs). (B) The fusion index [FI = (number of nuclei from total osteoclasts/nuclei of total cells) ×100%] of *Ads*-knockdown cells markedly decreased (FI =0) compared to the control *Luc*-knockdown cells (FI =41.40%) and untransfected control RAW264.7 cells (FI =26.11%). RANKL, receptor activator of nuclear factor-κB ligand.

**Figure 4:** Adseverin (*Ads*)-knockdown cells lack the ability to fuse even at high cell densities. Monocytes were plated at three initial plating densities, low (1×10^4^ cells/well), normal (5×10^4^ cells/well), and high (1×10^5^ cells/well), to observe the effects of cell density on osteoclastogenesis (OCG). Representative photomicrographs from *Ads*-knockdown and *Luc*-knockdown cultures are shown on days 0 and 4 of OCG, and representative TRAcP-stained images of day 4 cultures are shown on the right. At the 2-fold-higher normal plating density, *Ads*-knockdown cells cannot form more multinucleated osteoclasts, suggesting a fusion defect.

**Figure 5:** Adseverin (*Ads*) knockdown impaired RANKL-induced actin ring formation and bone resorption. (A) Actin rings were stained with Alexa 488-conjugated phalloidin. To visualize the nuclei, the cells were stained with 4′,6-diamidino-2-phenylindole (DAPI). Immunofluorescence images of osteoclast actin rings were visualized using confocal microscopy. *Ads*-knockdown cells have defective actin ring formation compared to *Luc*-knockdown cells. (C) The total number of rings/slide was counted. *Luc*-knockdown cells formed ~50 actin rings/field with clear and dense margins, whereas *Ads*-knockdown cells never formed actin rings.(B) *Ads*-knockdown and *Luc*-knockdown Raw264.7 cells stimulated with 60 ng/ml sRANKL were seeded onto dentin slices. On day 4, resorption pits formed on dentin slices were stained with 1% (w/v) toluidine blue. *Ads*-knockdown osteoclastic cultures had virtually no multinucleated osteoclasts on dentin disks (data not shown), and extremely small, seldomly-detected resorption pits. (D and E) The number and area of resorption pits were measured using ImageJ software. Results are expressed as the total area resorbed per dentine disc and the number of resorption pits. *Luc*-knockdown cells were capable of resorbing the dentin disc substrate at significantly higher rates. RANKL, receptor activator of nuclear factor-κB ligand.

**Figure 6:** Adseverin (*Ads*) knockdown is associated with impaired RANK signaling. Signaling downstream of RANK was evaluated by nuclear factor-κB (NF-κB) and c-jun immunostaining on day 4 of osteoclastogenesis (OCG). NF-κB was activated in *Luc*-knockdown osteoclasts as shown by its exclusively nuclear distribution (arrows). The majority *Ads*-knockdown macrophages did not exhibit active NF-κB, as shown by its cytoplasmic distribution. *Luc* knockdown and *Ads* knockdown demonstrated activated nuclear c-jun, a transcription factor involved in RANK survival signaling in osteoclasts. RANK, receptor activator of nuclear factor-κB.

## References

[1] Miyamoto T, Suda T (2003). Differentiation and function of osteoclasts. Keio J Med.

[2] Roodman GD (1999). Cell biology of the osteoclast. Exp Hematol.

[3] Asagiri M, Takayanagi H (2007). The molecular understanding of osteoclast differentiation. Bone.

[4] Troen BR (2003). Molecular mechanisms underlying osteoclast formation and activation. Exp Gerontol.

[5] Tanaka S (2007). Signaling axis in osteoclast biology and therapeutic targeting in the RANKL/RANK/OPG system. Am J Nephrol.

[6] Akisaka T, Yoshida H, Inoue S, Shimizu K (2001). Organization of cytoskeletal F-actin, G-actin, and gelsolin in the adhesion structures in cultured osteoclast. J Bone Miner Res.

[7] Garbe AI, Roscher A, Schüler C (2012). Regulation of bone mass and osteoclast function depend on the F-actin modulator SWAP-70. J Bone Miner Res.

[8] Kuhn TB, Brown MD, Bamburg JR (1998). Rac1-dependent actin filament organization in growth cones is necessary for beta1-integrin-mediated advance but not for growth on poly-D-lysine. J Neurobiol.

[9] Qian Y, Zhong X, Flynn DC (2005). ILK mediates actin filament rearrangements and cell migration and invasion through PI3K/Akt/Rac1 signaling. Oncogene.

[10] Aspenström P, Fransson A, Saras J (2004). Rho GTPases have diverse effects on the organization of the actin filament system. Biochem J.

[11] Kulkarni S, Goll DE, Fox JE (2002). Calpain cleaves RhoA generating a dominant-negative form that inhibits integrin-induced actin filament assembly and cell spreading. J Biol Chem.

[12] Gremm D, Wegner A (2000). Gelsolin as a calcium-regulated actin filament-capping protein. Eur J Biochem.

[13] McLaughlin PJ, Gooch JT, Mannherz HG, Weeds AG (1993). Structure of gelsolin segment 1-actin complex and the mechanism of filament severing. Nature.

[14] Prochniewicz E, Zhang Q, Janmey PA, Thomas DD (1996). Cooperativity in F-actin: binding of gelsolin at the barbed end affects structure and dynamics of the whole filament. J Mol Biol.

[15] Sun HQ, Wooten DC, Janmey PA, Yin HL (1994). The actin side-binding domain of gelsolin also caps actin filaments. Implications for actin filament severing. J Biol Chem.

[16] Arai M, Kwiatkowski DJ (1999). Differential developmentally regulated expression of gelsolin family members in the mouse. Dev Dyn.

[17] Robbens J, Louahed J, De Pestel K (1998). Murine adseverin (D5), a novel member of the gelsolin family, and murine adseverin are induced by interleukin-9 in T-helper lymphocytes. Mol Cell Biol.

[18] Dabiri GA, Young CL, Rosenbloom J, Southwick FS (1992). Molecular cloning of human macrophage capping protein cDNA. A unique member of the gelsolin/villin family expressed primarily in macrophages. J Biol Chem.

[19] Archer SK, Behm CA, Claudianos C, Campbell HD (2004). The flightless I protein and the gelsolin family in nuclear hormone receptor-mediated signalling. Biochem Soc Trans.

[20] McGough AM, Staiger CJ, Min JK, Simonetti KD (2003). The gelsolin family of actin regulatory proteins: modular structures, versatile functions. FEBS Lett.

[21] Pellieux C, Desgeorges A, Pigeon CH (2003). Cap G, a gelsolin family protein modulating protective effects of unidirectional shear stress. J Biol Chem.

[22] Sakurai T, Kurokawa H, Nonomura Y (1991). Comparison between the gelsolin and adseverin domain structure. J Biol Chem.

[23] Maekawa S, Sakai H (1990). Inhibition of actin regulatory activity of the 74-kDa protein from bovine adrenal medulla (adseverin) by some phospholipids. J Biol Chem.

[24] Maekawa S, Toriyama M (1994). Purification of tropomyosin from bovine adrenal medulla and its inhibitory effect on the actin severing activity of adseverin (adrenal medulla 74 kDa actin severing protein). Biochem Mol Biol Int.

[25] Nakamura S, Sakurai T, Nonomura Y (1994). Differential expression of bovine adseverin in adrenal gland revealed by in situ hybridization. Cloning of a cDNA for adseverin. J Biol Chem.

[26] Lueck A, Brown D, Kwiatkowski DJ (1998). The actin-binding proteins adseverin and gelsolin are both highly expressed but differentially localized in kidney and intestine. J Cell Sci.

[27] Chellaiah M, Kizer N, Silva M, Alvarez U, Kwiatkowski D, Hruska KA (2000). Gelsolin deficiency blocks podosome assembly and produces increased bone mass and strength. J Cell Biol.

[28] Wang Q, Xie Y, Du QS (2003). Regulation of the formation of osteoclastic actin rings by proline-rich tyrosine kinase 2 interacting with gelsolin. J Cell Biol.

[29] Beaulieu V, Da Silva N, Pastor-Soler N (2005). Modulation of the actin cytoskeleton via gelsolin regulates vacuolar H^+^-ATPase recycling. J Biol Chem.

[30] Yang G, Zaidi M, Zhang W (2008). Functional grouping of osteoclast genes revealed through microarray analysis. Biochem Biophys Res Commun.

[31] Wang Y, Belsham DD, Glogauer M (2009). Rac1 and Rac2 in osteoclastogenesis: a cell immortalization model. Calcif Tissue Int.

[32] Riedl J, Crevenna AH, Kessenbrock K (2008). Lifeact: a versatile marker to visualize F-actin. Nat Methods.

[33] Teitelbaum SL (2000). Bone resorption by osteoclasts. Science.

[34] Nurminsky D, Magee C, Faverman L, Nurminskaya M (2007). Regulation of chondrocyte differentiation by actin-severing protein adseverin. Dev Biol.

[35] Svensson C, Lundberg K (2001). Immune-specific up-regulation of adseverin gene expression by 2,3,7,8-tetrachlorodibenzo-p-dioxin. Mol Pharmacol.

[36] Svensson C, Silverstone AE, Lai ZW, Lundberg K (2002). Dioxin-induced adseverin expression in the mouse thymus is strictly regulated and dependent on the aryl hydrocarbon receptor. Biochem Biophys Res Commun.

[37] Iqbal J, Sun L, Cao J (2013). Smoke carcinogens cause bone loss through the aryl hydrocarbon receptor and induction of Cyp1 enzymes. Proc Natl Acad Sci USA.

[38] Vitale ML, Rodriguez Del Castillo A, Tchakarov L, Trifaró JM (1991). Cortical filamentous actin disassembly and scinderin redistribution during chromaffin cell stimulation precede exocytosis, a phenomenon not exhibited by gelsolin. J Cell Biol.

[39] Marcu MG, Rodriguez del Castillo A, Vitale ML, Trifaró JM (1994). Molecular cloning and functional expression of chromaffin cell scinderin indicates that it belongs to the family of Ca(2+)-dependent F-actin severing proteins. Mol Cell Biochem.

[40] Ehre C, Rossi AH, Abdullah LH (2005). Barrier role of actin filaments in regulated mucin secretion from airway goblet cells. Am J Physiol Cell Physiol.

[41] Shilagardi K, Li S, Luo F (2013). Actin-propelled invasive membrane protrusions promote fusogenic protein engagement during cell-cell fusion. Science.

[42] Taylor LM, Tertinegg I, Okuda A, Heersche JN (1989). Expression of calcitonin receptors during osteoclast differentiation in mouse metatarsals. J Bone Miner Res.

[43] Ikeda F, Matsubara T, Tsurukai T, Hata K, Nishimura R, Yoneda T (2008). JNK/c-Jun signaling mediates an anti-apoptotic effect of RANKL in osteoclasts. J Bone Miner Res.

